RETRACTED

# Analysis of Psychological Changes and Intervention Mechanism of Elderly Groups Based on Deep Learning Analysis Technology

**DOI:** 10.1155/2022/1686219

**Published:** 2022-04-30

**Authors:** Yue Gao, Qi Fan

**Affiliations:** ^1^Department of Psychology, School of Medicine & Holistic Integrative Medicine, Nanjing University of Chinese Medicine, Nanjing 210023, China; ^2^Institute of Mental Health, Nanjing Xiaozhuang University, Nanjing 210017, China

## Abstract

The elderly group is a unique social phenomenon in China. This study analyzes the typology of psychological changes in the elderly group based on the analysis of deep learning techniques and also combines crisis intervention theory to study the intervention strategies of social workers in different stages of emotional changes in the elderly group. A questionnaire survey of the elderly was conducted using the survey method, in which 10,948 valid questionnaires were screened from the Psychological Condition Self-check Scale and 11,040 valid questionnaires were screened from the Mental Health Survey Questionnaire for the Elderly. The degree of negative emotions of the elderly group in public emergencies was not related to age, but significantly correlated with age (*p* value < 0.05), and there was a tendency that the higher the age, the deeper the degree; in addition, elderly people of different professions also showed significant differences (*p* < 0.05); elderly people of different regions also showed significant differences (*p* < 0.05). In crisis intervention, social workers mainly provide services such as initial diagnosis, primary intervention, secondary intervention, and assessment for the caseworkers. The practical study found that social workers need to use strategies such as short-term focal solutions, avoiding guiding clients with their own values; crisis intervention programmes should be flexible, proactively helping clients to rebuild their support network, developing clients' self-solving skills, and implementing interprofessional teamwork and whole-person rehabilitation services.

## 1. Introduction

As the first generation of only-child parents move into old age, more and more problems are emerging for the elderly parents of only children. According to some scholars, nearly 100 million only child have been born in China over the past 30 years [1]. Most of the young couples who responded strictly to the national family planning policy and had only one child are now in their middle and old age. If they lose their only child, they become China's new generation, the “lost generation” [2]. Although there are no official statistics on the number of older people, demographic survey data and reports show that the number of older people is increasing and cannot be ignored. As they are past their child-bearing years, many of them are facing great trauma, with problems such as the breakdown of their family of origin and the inadequacy of the social security system causing them to suffer both physical and psychological blows, and they may face problems such as “no one to rely on, no one to turn to, no one to defend their rights, no one to interact with, no one to seek medical treatment for their illness, no one to support them in their old age, and no one to send them to their death” [3].

RETRACTED

At present, both the government and civil society are still not paying enough attention to this group. Social workers can, to a certain extent, help this group to effectively integrate multiple resources, repair the broken social network, and rebuild social support, thus restoring and enhancing their ability to adapt to their environment [4].

There are three main perspectives in the study of older people in China. One is the study of the number and growth trend, which is a macrolevel study by scholars, but lacks consideration of the microlevel of the single-parent group [5]. The second is the perspective of family-planning policy risks, where scholars have mainly explored the interrelationship between family planning policies, but lacked research on practical services for different family risks [6]. Thirdly, from the perspective of research on protection mechanisms, academics have studied the issue of social assistance for older people at the external levels of material and spirituality, but not enough research has been conducted on crisis interventions for older people to cope with risks and their ability to live independently [7]. Crisis intervention aims to help older people deal with emotional crises that they cannot cope with, provide them with social resources to avoid further harm, and help them return to the good state they were in before the crisis, in the process promoting their growth and improving their ability to cope [8]. Overseas research on the problems associated with only children focuses on the education and psychological aspects of growing up as an only child and comparisons with non-only children, but little research has been conducted on the issue of “lost children.” In addition, children need to become self-reliant as adults and are thus removed from the parental relationship [9]. In response to the lack of research on practical interventions for older people, this study attempts to answer the following questions: what are the aspects of the emotional crisis of older people, what are the practical theoretical foundations of crisis intervention, how to apply crisis intervention theory in the process of serving older people, what are the strategies and techniques of crisis intervention, how to reflect on the practice of crisis intervention, and so on [10].

RETRACTED

The elderly population is a special group that is easily affected during major public emergencies. The primary reason for this is that the elderly population is in a stage of rapid physical and mental development and change, with a high degree of instability; secondly, as the lifestyle of the elderly is inclined towards cerebral activities, their inner world has a relatively complex. Thirdly, as the lifestyle of older people is inclined towards mental activities, their inner world has a relatively complex nature [11]. As a result, the overall psychological needs of older people are high and may lead to psychological crises in times of social change, family conflicts, and setbacks in personal development [12]. As a result, the psychological crisis of the elderly population is the most important issue in the event of a major public emergency. The increasingly fierce competition in contemporary society and the gradually accelerating pace of life are bound to have an impact on the academic life of older people [13]. From a historical perspective, the great abundance of material conditions means that people will gradually face less stress in life and have less capacity to cope with unexpected events. There are numerous contemporary cases of psychological crises among the elderly due to various problems, and universities are paying more and more attention to mental health education for the elderly [14]. Therefore, it is of great importance to establish a perfect psychological crisis intervention mechanism for the elderly, to cultivate a positive psychological concept among them, to provide them with correct mental health education, and to guide them to face possible psychological crises by using strong will qualities, appropriate achievement motivation, and correct attribution methods, both for maintaining the life safety of the elderly and for building a harmonious society [15].

## 2. Practical Theory of Emotional Crisis Intervention for the Elderly

### 2.1. Theoretical Foundations

Lindemann, one of the founders of crisis theory, began with his study of the grief reactions of refugees and families of those who died in the Boston fire of 1943 and divided crisis intervention into four stages [16]: disruption of equilibrium, short course therapy or grief intervention for the client, overcoming the crisis or coming out of discomfort, and regaining equilibrium (see Figure 1).

This theory suggests that the longer an older person is in a state of severe depression, especially in bereavement, the higher the risk of falling into excessive grief, leading to a loss of balance and a state of crisis. The social worker should help the client to get out of the emotional crisis as soon as possible by giving them adequate support and linking them to resources to restore their pre-crisis state of equilibrium [17].

RETRACTED

The Kubler–Ross model, which describes the emotional reactions that people experience when facing their impending death, has since been widely applied to the study of grief following the loss of a loved one.  Figure 2 shows the extended crisis theory model.

First is the period of denial. When people hear news of a terminal illness or death of themselves or a family member, they will first feel shocked and numb and psychologically deny the truth of the information they receive about the death. Second is the period of anger. After the shock and numbness have passed, the case worker becomes very angry, lashing out at those around him or her and blaming himself or herself or others for the death. Third is the bargaining period. During this period, the caseworker enters a period of self-deception, hoping for another chance to make up for what was not accomplished in the past. The caseworker will bargain with God for a series of things in exchange for or to prolong life. Fourth is the depression phase. During this phase, the caseworker has two depressive tendencies, reactive depression, which is an ineradicable emotional reaction, and preparatory depression, which is an internal emotional preparation to give up on everything. Fifth is the period of acceptance. After going through the whole grief journey, the caseworker begins to accept the status quo and shows a state of calmness, but this phase is the most melancholic period.

As with bereavement in general, older people who have lost someone go through this series of emotional changes, but not everyone will go through every stage, some will skip certain stages and some will stay at a certain stage. Older people who have lost someone may take longer to move through each stage of emotional change than at other ages or other bereavement events.

Without grief counselling from professionals, it can be difficult for the bereaved elderly to get out of their situation on their own. Moreover, feelings of self-blame and irrational emotions will be more pronounced in the elderly who have lost a parent, and the worse their physical and mental state, the greater the likelihood of depression.

### 2.2. Support Network Rupture and Reconstruction: A Case Intervention in an Emotional Crisis

Crisis assessment requires the identification of the client's crisis situation, the planning of crisis intervention services, and a specific diagnosis of post-traumatic stress disorder [18]. The assessment is generally done in a funnel style, moving from an assessment of the client's wider social environment to a focused assessment of the core issues, which is a subjective and uncertain process (see Figure 3).

RETRACTED

This case is an emotional crisis and a developmental crisis. Through crisis management strategies, the social worker helped the client to cope with the internal or external stress caused by the loss of her son (see Figure 4). In the intervention, the principles of immediate response, time limitation, focus on the crisis structure, problem solving, self-determination of the client, and social network connection were followed.

## 3. Modelling Mental Health Status Calculations

### 3.1. Data Collection

This study used a self-developed online experiment platform to collect data from Sina Weibo users (Figure 5). During April 2012, a total of 563 Sina Weibo users volunteered to participate in the experiment. In order to ensure a sufficient amount of online data for the subjects, active users were selected from the recruited users with requirement that they had posted at least 500 tweets before the experiment and that the latest tweet was posted within 3 months before the experiment, thus effectively eliminating inactive users from the data. In order to ensure the quality of the psychological characteristics of the subjects, the subjects were required to fill in the online psychological questionnaire according to the standard. In this study, subjects who failed to answer the questionnaire were excluded [19]. After the screening process, 444 subjects (171 males and 273 females, average age 23.8 years old) remained, and their education level was mainly undergraduate (43%) and college (24%). The monthly per capita disposable income of the subjects was concentrated in the range of 1000–2000 RMB (25%) and 2000–5000 RMB (22%). Data from eligible subjects were used for subsequent model training.

### 3.2. Data Measurement

#### 3.2.1. Mental Health Status

In this study, the Symptom Checklist 90 (SCL-90) [20] was used to measure the depression and anxiety levels of the subjects. The SCL-90 is a widely used international instrument for measuring mental health status, with good reliability and validity [21]. The questionnaire consists of a series of mental health symptoms, and subjects are asked to rate the severity of each mental health symptom on a 5-point Likert-type scale (0 being never and 4 being severe). The number of questions measuring depression and anxiety was 13 and 10, respectively, with higher scores indicating more severe mental health problems.

RETRACTED

#### 3.2.2. Online Behavioural Characteristics

In this study, based on the common types of online behavioral characteristics, we designed four categories of online behavioral characteristics based on the functions and data format of Sina Weibo, and the characteristics of the modeling target (mental health status). Based on the features of Sina Weibo, we designed 45 online behavioral characteristics in 4 categories [22]. Among them, (1) user information features describes the basic personal information of the subjects (e.g., gender and place of origin), (2) self-presentation features describe how the subjects create a virtual personal image on the online platform and present it to other users (e.g., whether to use the system's default virtual avatar), (3) privacy settings' features describe the subjects' preferences for personal privacy protection (e.g., whether to allow strangers on their personal pages), (4) privacy settings' features describe the subjects' preferences for privacy protection (e.g., whether to allow strangers on their personal pages), and (5) social network characteristics describe subjects' interpersonal interactions on online platforms (e.g., number of “followers” and number of “mutual followers”). For the Boolean features, they were binary coded, while for the floating-point features, the original values were retained.

### 3.3. Data Modeling

Mental health includes a range of different mental health dimensions (e.g. depression and anxiety), which are related to each other to a certain extent. The effectiveness of data modeling can be improved if common information between different mental health dimensions is taken into account when building a computational model for a specific mental health dimension.

The basic idea of the multitask regression approach is that there are assumed to be *T* tasks and N instances, each with a training dataset {(*x*_*tn*_, *y*_*tn*_)}(*t*=1,2,…, *T*; *n*=1,2,…, *N*). Each instance can be represented as x⊆Rd and y⊆RT (with feature number *d*) and matched with a multidimensional output vector (e.g., depression and anxiety dimensions), with the aim of finding a *T* × *d* matrix of coefficients, e.g.,

(1) $$\begin{array}{c} W=\arg\min\left\{L\left(x,y,W;1:T\right)+\lambda \Omega \left(W\right)\right\}. \end{array}$$

In this study, L(x, y,W; 1 : T) is denoted as the empirical loss function, Ω(**W**) is denoted as the regularizer, and *λ* is denoted as the tradeoff constant [23]. In this study, L(x, y,W; 1 : T) is set as the least square error, and Ω(**W**) is set as the Frobenius norm. That is,

(2) $$\begin{array}{c} L\left(x,y,W;1:T\right)=Y-\hat{Y}=\sum_{t=1}^{T}\sum_{n=1}^{N}{\left(y_{tn}-{\hat{y}}_{tn}\right)}^{2} \end{array}$$

(3) $$\begin{array}{c} \Omega \left(W\right)={\left\|W\right\|}^{2}=\text{tr}\left(W^{T}.W\right). \end{array}$$

Substituting (2) and (3) into equation (1), i.e.,

(4) $$\begin{array}{c} W={\left(\lambda I+\sum_{n}x_{n}x_{n}^{T}\right)}^{-1}\left(\sum_{n}x_{n}y_{n}^{T}\right). \end{array}$$

For the selection of *λ*, a bias-variance decomposition method was used to minimize the expected loss of [(error) +variance]. In view of this, the multitask regression method [24, 25] was used to develop models for depressive and anxiety states based on network data analysis. This study also used linear regression and feedforward neural network to develop the same mental health state model, which was used as a baseline model to evaluate the effectiveness of the multitask regression method.

RETRACTED

## 4. Study Results

After tuning the model parameters, the learning rate of the feedforward neural network method was set to 0.9 and the parameter *λ* of the multitask regression method was set to 1.70 (ln (*λ*)=0.53). The correlation coefficients between the results of the mental health state model and the psychological questionnaire are shown in Table 1, and the network behavioral characteristics that were significantly correlated with depression and anxiety are shown in Table 2. For the same modeling target (depression or anxiety), the results of the mental health state model based on different modeling methods were different [26]. It is noteworthy that the correlation coefficient between the results of the mental health state model and the results of the psychological questionnaire was the highest among the three different modeling approaches for both the depression and anxiety dimensions.

Analysis of the data showed no significant gender differences in anxiety and depression during major public events, anxiety *t* = -0.865, *p* = 0.387; depression *t* = -0.011, and *p* = 0.991; but regionally, significant differences were shown, anxiety *F* (31, 10 916) = 1.713, *p* = 0.008, and depression *F* (31, 10 916) = 3.687, *p* = 0.000; unexpectedly, the region with the highest levels of both anxiety and depression among older people was Guangxi (M (anxiety) = 9.38, SD = 3.264, and *M* (depression) = 12.05, SD = 4.011). The data showed that the levels of anxiety and depression among older people in this major public event differed between groups of older people, with anxiety *F*9,10 938) = 3.757, *p* = 0.000, and depression *F*(9,10 938) = 3.840, *p* = 0.000, and the differences were highly significant. It is noteworthy that there were no significant differences in anxiety and depression between ages, but there were significant differences between ages, with anxiety *F* (2, 10 945) = 5.495, *p* = 0.004, and depression *F* (2, 10 945) = 5.117, *p* = 0.006, and it is easy to see from the images that, as age increases, the levels of anxiety and depression caused by major public events The degree of anxiety and depression due to major public events increased significantly and linearly with age, see Figure 6.

RETRACTED

However, significant age differences were found in only some of the older adult groups. Again, not all regions showed significant age differences, with the most significant differences being in Inner Mongolia, where *F* (2, 1,147) = 5.221, *p* = 0.006, and in depression, *F* (2, 1,147) = 4.997, *p* = 0.007. Anxiety was *F* (2, 231) = 3.966, *p* = 0.020, and depression was *F* (2, 231) = 6.034, *p* = 0.003.

The analysis of the results of the mental health questionnaire for older people showed results that were largely consistent with the results of the Psychological Status Self-Assessment Scale [27]. There were no significant differences in total questionnaire scores by age, but there were significant differences by age, *F* (2, 11,037) = 4.916, *p* = 0.007. Tests of variance for each dimension of the Psychological Screening Questionnaire for Older People showed that the most significant differences between ages were for life events, followed by social support and personality traits, see Table 3.

## 5. Conclusions

By collating and analysing the results of psychological assessments conducted on older people through big data, we can accurately identify groups with potential psychological crises and develop psychological support programmes to promote psychological resources to groups in greater need, which is of great guidance in helping counsellors to complete psychological crisis screening, effectively improve the timeliness of psychological counselling work, and improve the directionality of psychological support and psychological construction. Combined with the results of big data analysis, the construction of a complete psychological crisis intervention system will help to give full play to the important role of cadres and counsellors of the elderly, form a four-level crisis prevention and intervention system of schools, psychological centres, counsellors of elderly groups, and class-level psychological members, monitor the psychological dynamics of the elderly in real time, carry out psychological health education, improve the response rate when facing psychological crises, and effectively help the elderly cope with potential psychological crises arising from major emergencies.

## Figures and Tables

**Figure 1:** Lindemann crisis theory model.

RETRACTED

**Figure 2:** Extended crisis theory model.

**Figure 3:** Hierarchy of prognosis in a funnel.

**Figure 4:** Ecological map of the case owner's family.

**Figure 5:** Subject data collection process.

**Figure 6:** Comparison of psychological profiles between ages.

**Table 1:** Calculated results of the mental health state model and the results of the psychological questionnaire: correlation coefficients between the results of the mental health model and the results of the psychological questionnaire.

	Linear regression	Feedforward neural network	Multitask regression
Depressed	0.12	0.26	0.41
Anxious	0.14	0.21	0.34

**Table 2:** Correlation coefficient values for selected online behavioural characteristics and mental health dimensions.

Features	Depressed	Anxious
Gender	−0.137	−0.148
Original “microblog” ratio	−0.085	−0.094
Screen name length	0.166	0.073

**Table 3:** Test of variance for each dimension of the Older People's Mental Health Survey questionnaire.

Dimension	*F*	Sig
Growth experience	0.66	0.517
Personality traits	4.646	0.01
Life events	69.206	0
Social support	8.688	0

## Data Availability

The experimental data used to support the findings of this study are available from the corresponding author upon request.
